The article "Correlation between Levels of Serum Lipoprotein-Associated Phospholipase A2 and Soluble Suppression of Tumorigenicity 2 and Condition of Acute Heart Failure Patients and Their Predictive Value for Prognosis" was published in 2021. Journal: J Healthc Eng.

# Correlation between Levels of Serum Lipoprotein-Associated Phospholipase A2 and Soluble Suppression of Tumorigenicity 2 and Condition of Acute Heart Failure Patients and Their Predictive Value for Prognosis

**DOI:** 10.1155/2021/1525190

**Published:** 2021-12-16

**Authors:** Jinjin Zhang, Lei Wang, Zhikun Zhao, Liang Li, Yunfeng Xia

**Affiliations:** Department of Geriatric Medicine, The Fourth Medical Center of PLA General Hospital, Beijing, China

## Abstract

**Objective:**

To explore the correlation between levels of serum lipoprotein-associated phospholipase A2 (LP-PLA2) and soluble suppression of tumorigenicity 2 (sST2) and condition of acute heart failure (AHF) patients and their predictive value for prognosis.

**Methods:**

The data of patients who complained of acute dyspnea and were treated in our hospital (January 2018–January 2020) were selected for review analysis, and those diagnosed with AHF by means of chest films, physical examination, cardiogram, and color Doppler ultrasonography (CDS) were selected as the study objects. The patients were split into the mild group (I or II, 55 cases) and the severe group (III or IV, 50 cases) according to the clinical condition grading standard in *Guidelines for Diagnosis and Treatment of Acute Heart Failure*. In addition, 105 healthy individuals examined in our medical center in the same period were selected as the control group. The serum LP-PLA2 and sST2 levels of all study objects were measured to analyze the correlation between these levels and AHF condition. Readmission due to heart failure and all-cause death were regarded as the endpoint events, and after one year of follow-up visits, the occurrence of the endpoint events in patients of the two groups was recorded, and with the endpoint events as the variable, the patients were divided into the event group and nonevent group to establish a logistic regression analysis model and analyze the merit of serum LP-PLA2 and sST2 in evaluating patient outcome.

**Results:**

The patients' general information such as age and gender between the severe group and the mild group were not statistically different (*P* > 0.05), and the levels of high-sensitivity c-reactive protein (CRP), hemoglobin, creatinine, and uric acid of the severe group were greatly different from those of the mild group (*P* < 0.001), the comparison result of serum LP-PLA2 and sST2 levels was severe group > mild group > control group (*P* all <0.001), and the serum LP-PLA2 and sST2 levels of the severe group were, respectively, 275.98 ± 50.68 ng/ml and 2,122.65 ± 568.65 ng/ml; among 105 AHF patients, 50 of them had endpoint events (47.6%), including 36 in the severe group (36/50, 72.0%) and 14 in the mild group (14/55, 25.5%), and the event group presented greatly higher serum LP-PLA2 and sST2 levels than in the nonevent group (*P* < 0.001); according to the logistic regression analysis, serum LP-PLA2 and sST2 had independent predictive value for prognosis of AHF patients, which could be used as the independent predictive factors for 1-year prognosis.

The article "Correlation between Levels of Serum Lipoprotein-Associated Phospholipase A2 and Soluble Suppression of Tumorigenicity 2 and Condition of Acute Heart Failure Patients and Their Predictive Value for Prognosis" was published in 2021. Journal: J Healthc Eng.

**Conclusion:**

Serum LP-PLA2 and sST2 have a good diagnosis value for the condition and prognosis of AHF patients, which shall be promoted and applied in practice.

## 1. Introduction

Being a kind of clinical syndrome that endangers patients' lives, acute heart failure (AHF) refers to sudden heart failure (HF) or aggravation of the original HF signs, and AHF patients clinically show a significant decrease in cardiac contractility, a marked increase in cardiac workload, a sudden decline in cardiac output, and a dramatic rise in the pulmonary circulation pressure, which consequently triggers symptoms such as pulmonary congestion, pulmonary edema, and cardiogenic shock [1, 2]. According to data from the European ESC-HF study, the rate of all-cause death within 1 year was 24.0% in AHF patients, and the 3-year and 5-year mortality rates were as high as 30.0% and 60.0% of in-patients with heart failure [3]; among 3,335 AHF patients prospectively registered at 14 hospitals in Beijing, 15% of them died within 30 d and 32.3% died at 1 year, and the patient death or readmission rate was as high as 60.0% [4], indicating that despite improved diagnosis and treatment of AHF, the short-term and long-term patient prognosis are still not promising. Nowadays, the incidence of AHF is rising enormously with the worldwide aging [5], the prevalence is above 10.0% in those aged over 70 years, and the number of patients who die from the disease is also increasing. From a practical point of view, further analyzing the severity and risk grading of AHF in patients with objective tools to improve treatment level and effectively evaluate patient prognosis is now the focus of clinical investigation.

Recently, significant progress has been made in the diagnosis of serum markers, and some serum markers are confirmed to be closely related to the prognosis of HF [6, 7]. Since ventricular remodeling is a key element affecting the prognosis of HF patients, suppression of tumorigenicity 2 (ST2) in humans, which is related to the pathophysiology of ventricular remodeling, has been identified as an important indicator for assessing the prognosis of chronic HF (CHF) patients, and most studies have shown that this substance can act through the IL-33/ST2 pathway in the development and progression of HF [8, 9]. SST2 is the soluble ST2, and the PRIDE study demonstrated a positive association between sST2 levels and symptom severity by NYHA Functional Classification and that sST2 level was an independent factor for predicting the risk of mortality from acute dyspnea [10]. In addition to sST2, the release of proinflammatory factors triggered by impaired endothelial cells in the arterial vessel wall aggravates ventricular remodeling as well, indicating that immune inflammatory activation is important in HF progression. Lipoprotein-associated phospholipase A2 (LP-PLA2) is an important inflammatory enzyme that leads to abnormal secretion of proinflammatory factors, and numerous epidemiological studies have shown that it is an independent predictor of cardiovascular events (CVEs), which can effectively assess the prognosis of cardiovascular disease (CVD) patients [11, 12]. Currently, LP-PLA2 and sST2 are mostly used in studies on CHF [13], but there is no literature systematically exploring the value of both for the assessment and prediction of AHF. Based on this, the relationship between serum LP-PLA2 and sST2 levels and AHF condition and the predictive value for prognosis were investigated herein, which is reported as follows.

The article "Correlation between Levels of Serum Lipoprotein-Associated Phospholipase A2 and Soluble Suppression of Tumorigenicity 2 and Condition of Acute Heart Failure Patients and Their Predictive Value for Prognosis" was published in 2021. Journal: J Healthc Eng.

## 2. Data and Methods

### 2.1. Study Design

This review study was conducted in our hospital from January 2018 to January 2020 to investigate the relationship between serum LP-PLA2 and sST2 levels and AHF condition and their predictive value for prognosis.

### 2.2. Blinding Level

It was a double-blind study; i.e., neither the research objects nor researchers understood the trial grouping, and the study designer was responsible for arranging and controlling the full trial.

### 2.3. Enrollment of Research Objects

The data of patients who complained of acute dyspnea and were treated in our hospital from January 2018 to January 2020 were selected for review analysis, and the patients were enrolled by the following criteria. Inclusion criteria: (1) patients' signs, chest films, electrocardiograms (ECGs), and cardiograms met the AHF diagnosis criteria in *Guidelines for Diagnosis and Treatment of Acute Heart Failure* [14]; (2) their medical records were complete. Exclusion criteria: (1) the patients could not communicate with others because of factors such as mental disturbance and communication disorders; (2) the patients quit the trail in the middle of treatment (including all kinds of reasons) or were lost to follow-up; (3) the patients had combined malignant tumor, primary gout, hematological disease, immune disease, end-stage renal disease, and thyroid dysfunction; and (4) the patients had combined intracranial or systemic infection.

The article "Correlation between Levels of Serum Lipoprotein-Associated Phospholipase A2 and Soluble Suppression of Tumorigenicity 2 and Condition of Acute Heart Failure Patients and Their Predictive Value for Prognosis" was published in 2021. Journal: J Healthc Eng.

### 2.4. Grouping Standard

In the study, 105 patients were enrolled and split into the mild group (I or II, 55 cases) and severe group (III or IV, 50 cases) according to the clinical condition grading criteria in the *Guidelines for Diagnosis and Treatment of Acute Heart Failure*; in addition, 105 healthy individuals examined in our medical center in the same period with no medical history of myocardial infarction and heart failure were selected as the control group.

### 2.5. Moral Consideration

The study met the principles in *World Medical Association Declaration of Helsinki* (2013) [15]. After enrollment, the study team explained the study purpose, meaning, contents, and confidentiality to the patients and asked the patients to sign the informed consent.

## 3. Methods

### 3.1. Collecting Clinical Data

On the day that the patients were enrolled, their clinical data were collected to establish a basic database, including (1) admission time, name, age, gender, contact information, height, body mass, and body mass index (BMI); (2) chief complain, admission diagnosis, and heart function, heart rate, and blood pressure at admission; (3) medical history of valvular heart disease, hypertension, diabetes, coronary heart disease (CHD), congestive HF, etc.; and (4) data of routine examinations at admission, including the routine blood test, blood biochemical examination, blood gas analysis, myocardial injury, cardiac function markers, and serum LP-PLA2 and sST2.

### 3.2. Processing Blood Samples

1. Serum collection of the control group: the peripheral blood was drawn from 105 healthy individuals and centrifuged under 2,000 r/min for 20 min to extract the supernatant for preservation, and their serum LP-PLA2 and sST2 levels were measured by the ELISA method (Beijing Kewei Clinical Diagnostic Reagent Inc.; NMPA approval no. S20060028)
2. Serum collection of patients: within 2 h after admission, the peripheral venous blood of 105 patients was drawn and centrifuged under 2,000 r/min for 20 min to extract the supernatant for preservation, and their serum LP-PLA2 and sST2 levels were measured in the same way as above

### 3.3. Follow-Up Visit

One-year follow-up was conducted for those in the severe group and the mild group to determine the changes in their clinical condition, if their symptoms such as chest distress, dyspnea, and fatigue were ameliorated, lung rales were reduced or fluid retention was improved, and it was considered as an improvement of the disease, and vice versa. In case of all-cause death or readmission due to heart failure, it was determined that adverse cardiac events (endpoint events) occurred, and the numbers of patients with endpoint events were recorded.

The article "Correlation between Levels of Serum Lipoprotein-Associated Phospholipase A2 and Soluble Suppression of Tumorigenicity 2 and Condition of Acute Heart Failure Patients and Their Predictive Value for Prognosis" was published in 2021. Journal: J Healthc Eng.

### 3.4. Observation Criteria

1. General information: the patients' general information were compared between the two groups
2. Analysis on the correlation between serum LP-PLA2 and sST2 levels and AHF condition: the levels of patients at admission were compared with the healthy individuals of the control group
3. Comparison of serum LP-PLA2 and sST2 levels between the event group and nonevent group: the numbers of patients with endpoint events in the severe group and the mild group one year later were counted, and with endpoint events happening in AHF patients as the basis, AHF patients were divided into the event group and the nonevent group, and their serum LP-PLA2 and sST2 levels were compared
4. Analysis on the efficacy of determining patient prognosis with serum LP-PLA2 and sST2: a logistic regression analysis model was established to analyze the efficacy of determining patient prognosis with serum LP-PLA2 and sST2

### 3.5. Statistical Processing

In this study, the data processing software was SPSS20.0, the picture drawing software was GraphPad Prism 7 (GraphPad Software, San Diego, USA), the items included were enumeration data and measurement data, which were examined by the *X*^2^ test and *t*-test, respectively, and differences were considered statistically significant at *P* < 0.05.

## 4. Results

### 4.1. General Information

No between-group statistical differences in patients' general information such as age and gender were observed (*P* > 0.05), and the levels of high-sensitivity C-reactive protein (CRP), hemoglobin, creatinine, and uric acid of the severe group were remarkably different from those of the mild group (*P* < 0.001), see Table 1.

### 4.2. Analysis on the Correlation between Serum LP-PLA2 and sST2 Levels and AHF Condition

Among the severe group, mild group, and control group, the comparison result of serum LP-PLA2 and sST2 levels was severe group > mild group > control group (*P* all <0.001), see Figure 1.

### 4.3. Comparison of Serum LP-PLA2 and sST2 Levels between the Event Group and the Nonevent Group

Among 105 AHF patients, a total of 50 cases (47.6%) had endpoint events, including 36 in the severe group (36/50, 72.0%) and 14 in the mild group (14/55, 25.5%), and the serum LP-PLA2 and sST2 levels were greatly higher in the event group than in the nonevent group (*P* < 0.001), see Figure 2.

### 4.4. Analysis on the Efficacy of Determining Patient Prognosis with Serum LP-PLA2 and sST2

According to the logistic regression analysis, serum LP-PLA2 and sST2 had independent predictive value for prognosis of AHF patients and could be used as the independent predictors for 1-year patient prognosis, see Table 2.

The article "Correlation between Levels of Serum Lipoprotein-Associated Phospholipase A2 and Soluble Suppression of Tumorigenicity 2 and Condition of Acute Heart Failure Patients and Their Predictive Value for Prognosis" was published in 2021. Journal: J Healthc Eng.

## 5. Discussion

AHF is defined as the acute exacerbation or sudden onset in a patient with CHF, which presents clinically as either systolic or diastolic HF, with the majority of patients experiencing clinical symptoms such as fatigue, acute dyspnea, and gasping. After systemic treatment, AHF patients are still vulnerable to recurrent HF, and some of them even face mortality outcomes, resulting in not promising prognosis. Data from recent years have shown an increasing trend of mortality within 1 year after discharge in AHF patients, and the rate of all-cause mortality is higher than 36.0% in Japan [16]. On this basis, assessing patient prognosis to reduce the risk of death with the help of objective tools has become a clinical hot spot. At this stage, based on different research ideas, a variety of biomarkers have been confirmed to be strongly linked to the incidence and progression of AHF [17, 18]. This study centered on immune inflammation because a large number of studies have shown that immune inflammation activation plays a crucial role in triggering and promoting HF [19]. When body immune inflammation is activated in HF patients, whether it is the long-term chronic inflammatory response in CHF patients or the sudden increase of inflammatory factors in AHF patients, immune inflammation can accelerate ventricular remodeling, leading to gradually aggravated myocardial injury and further deteriorated cardiac function, so it could predict the prognosis of HF patients to some extent.

In general, immune inflammation indicators are mostly used in the evaluation of CHF, but recent studies have shown that they are also tightly associated with the prognosis of AHF patients [20]. According to the report by scholar Mehmood Muddassir, AHF patients with a higher level of inflammation had an increased rate of in-hospital mortality [21], suggesting that inflammation indicators were related to the condition of AHF, and thus, factors inducing inflammation could be used to evaluate patient prognosis.

Recently, LP-PLA2 is a new-found inflammatory enzyme, which is a key factor to trigger imbalance of the inflammatory factor network and able to hydrolyze oxidized lecithin on arterial intima, allowing it to produce lysophospholipid choline and oxidized fatty acids, both of which can secrete large amounts of proinflammatory substances after chemotaxing inflammatory cells and then accelerate ventricular remodeling. A large number of epidemiological trials have shown that LP-PLA2 is an independent factor for predicting CVE [22]. Scholars Xiong et al. corrected the risk factors of traditional CVD and found that LP-PLA2 was still a risk predictor for CVE and had a positive correlation with the severity of CHF; e.g.,, the elevated level of CHF could increase the LP-PLA2 level [23]. In this study, no statistical differences in the enrolled patients' general information such as age and gender were observed (*P* > 0.05), the serum LP-PLA2 levels were obviously different between the severe group and the mild group, and according to the logistic regression analysis, serum LP-PLA2 had independent predictive value for AHF prognosis, demonstrating that its level was of great importance in AHF and not just in CHD and CHF.

The article "Correlation between Levels of Serum Lipoprotein-Associated Phospholipase A2 and Soluble Suppression of Tumorigenicity 2 and Condition of Acute Heart Failure Patients and Their Predictive Value for Prognosis" was published in 2021. Journal: J Healthc Eng.

Other than LP-PLA2, sST2 is also tightly linked to the immune inflammation. ST2, a member of the interleukin-1 receptor family, can combine with IL-33 to form the IL-33/ST2 signaling pathway and then promote HF progression. Early studies considered that ST2 was mainly involved in the immune inflammatory response through macrophages or T lymphocytes, and recent studies showed that it would exhibit an obvious upward trend when the heart was exposed to mechanical stretch stimuli, thereby competing for the binding site of ST2 to IL-33 and inhibiting the cardioprotective effect of the IL-33/ST2 signaling pathway [24, 25]. Therefore, elevated sST2 levels may be related to an increased risk of cardiovascular events. The study showed the comparison result of sST2 levels of severe group > mild group > control group (*P* all <0.001), indicating that the sST2 levels were obviously increased in AHF patients, and the more serious the HF, the higher the sST2 levels, implying that sST2 could be used to grade the AHF condition. After 1 year of follow-up visits, a total of 50 cases had endpoint events among the 106 patients (47.6%), including 36 in the severe group (36/50, 72.0%) and 14 in the mild group (14/55, 25.5%), and the serum LP-PLA2 and sST2 levels were remarkably higher in the event group than in the nonevent group (*P* < 0.001), denoting that sST2 was valuable in predicting prognostic events for AHF patients. In addition, according to the logistic regression analysis, it was proved that sST2 could be used as an independent predictor of 1-year patient prognosis with a better evaluation value, which could be jointly applied with LP-PLA2 in the evaluation of condition and prognosis of AHF patients.

To sum up, serum LP-PLA2 and sST2 have a good evaluation value for condition and prognosis of AHF patients, which shall be promoted and applied in practice.

## Figures and Tables

**Figure 1:** Serum indicators ($\bar{x}\pm s$, ng/ml). (a) The serum LP-PLA2 levels in ng/ml, and the comparison result was severe group > mild group > control group (275.98 ± 50.68 vs. 185.68 ± 45.68 vs. 165.22 ± 23.59, *P* all <0.001). (b) The serum sST2 levels in ng/ml, and the comparison result was severe group > mild group > control group (2,122.65 ± 568.65 vs. 1,568.65 ± 340.98 vs. 598.65 ± 110.68, *P* all <0.001). *Note.* In (a) and (b), the horizontal axes indicated the three groups (severe, mild and control) and # indicated *P* < 0.001.

The article "Correlation between Levels of Serum Lipoprotein-Associated Phospholipase A2 and Soluble Suppression of Tumorigenicity 2 and Condition of Acute Heart Failure Patients and Their Predictive Value for Prognosis" was published in 2021. Journal: J Healthc Eng.

**Figure 2:** Comparison of serum LP-PLA2 and sST2 levels between the event group and the nonevent group ($\bar{x}\pm s$, ng/ml). (a) The LP-PLA2 and sST2 levels of patients in the severe group, and the comparison result was event group > nonevent group (321.68 ± 45.85 vs. 265.98 ± 35.68, 2,598.65 ± 52.98 vs. 1,968.65 ± 368.65, *P* < 0.001). (b) The LP-PLA2 and sST2 levels of patients in the mild group, and the comparison result was event group > nonevent group (280.65 ± 35.65 vs. 172.65 ± 30.65, 2,125.65 ± 562.56 vs. 1,589.65 ± 350.58, *P* < 0.001). (c) The LP-PLA2 and sST2 levels of 105 AHF patients, and the comparison result was event group > nonevent group (294.65 ± 35.65 vs. 190.68 ± 15.68, 2,435.65 ± 568.98 vs. 1,148.65 ± 420.68, *P* < 0.001). *Note.* The horizontal axes indicated the event group and nonevent group; the black areas and gray areas, respectively, indicated LP-PLA2 and sST2; and # indicated *P* < 0.001.

**Table 1:** General information.

Group	Mild (*n* = 55)	Severe (*n* = 50)	*X* ^2^/*t*	*P*
Gender (male/female)	30/25	28/22	0.022	0.881
Age (years)	74.68 ± 2.65	74.99 ± 2.60	0.604	0.547
Mean body weight (kg)	60.69 ± 2.45	61.01 ± 2.85	0.618	0.538
BMI (kg/m^2^)	23.45 ± 1.20	23.57 ± 1.24	0.504	0.616
Height (cm)	173.65 ± 12.40	173.98 ± 11.68	0.140	0.889
*Medical history*				
Valvular heart disease	10	12	0.535	0.464
Hypertension	18	19	0.319	0.572
Diabetes	15	12	0.147	0.702
CHD	15	16	0.281	0.596
Congestive HF	10	8	0.088	0.767
LVEF (%)	50.55 ± 15.68	43.58 ± 15.40	2.294	0.024
High-sensitivity CRP (mg/L)	13.54 ± 4.68	28.65 ± 8.98	10.953	<0.001
Hemoglobin (g/L)	130.65 ± 8.99	122.98 ± 9.21	4.316	<0.001
Creatinine (*μ*mol/L)	95.62 ± 10.11	131.68 ± 12.35	16.431	<0.001
Uric acid (*μ*mol/L)	430.98 ± 56.32	489.65 ± 62.98	5.039	<0.001

**Table 2:** Analysis on the efficacy of determining patient prognosis with serum LP-PLA2 and sST2.

	B	S.E.	Wals	OR	Sig.	Exp (B)	Exp (B) 95% CI lower limit and upper limit	
LP-PLA2	0.000	0.000	4.568	1.001	0.036	1.000	1.000	1.001
sST2	0.002	0.001	14.756	1.002	0.000	1.002	1.000	1.003

## Data Availability

Data that support the findings of this study are available on reasonable request from the corresponding author.
